The article "The Prevalence of Neurological Complication after Renal Transplantation" was retracted in 2023. Reasons: unreliable results or conclusions; concerns about the data; concerns about the peer review; concerns about the citations.

# The Prevalence of Neurological Complication after Renal Transplantation

**DOI:** 10.1155/2022/8763304

**Published:** 2022-07-04

**Authors:** Xiaorong Zhu, Liangrong Shen, Dan Li, Luoning Shi, Qing Zhang

**Affiliations:** ^1^Department of Kidney Transplantation, The First Affiliated Hospital of Xi'an Jiaotong University School of Medicine, Xi'an, China; ^2^Disinfection Supply Center, The First Affiliated Hospital of Xi'an Jiaotong University School of Medicine, Xi'an, China; ^3^Department of Endocrinology, The First Affiliated Hospital of Xi'an Jiaotong University School of Medicine, Xi'an, China

## Abstract

**Objective:**

To evaluate the incidence of neurological complications (NCs) after renal transplantation by meta-analysis.

**Methods:**

A broad literature search in PubMed, Embase, and Cochrane-Library was performed from inception to December 31, 2021, to collect published studies on the incidence of NCs after kidney transplantation. The R language meta-package was used to organize and analyze the data.

**Results:**

17 articles including 1,1119 participants were considered eligible. There were 3 studies that recorded unclassified NCs (249 participants), 6 that recorded nervous system CMV infection (1489 participants), 3 that recorded headache (243 participants), and 5 that recorded cerebrovascular events (9138 participants). There was significant heterogeneity (all *I*^2^ ≥ 75%) in all analyses, and random-effects models were selected. Meta-analysis results showed that the incidence of unclassified NCs was 0.29 (95% CI (0.16–0.48)), the incidence of nervous system CMV infection was 0.38 (95% CI (0.26–0.52)), the incidence of headache was 0.55 (95% CI (0.44–0.66)), and the incidence of stroke was 0.05 (95% CI (0.02–0.09)). Egger's test showed that there was no conspicuous publication bias in the included literature in each group.

**Conclusions:**

Headache had the highest incidence (55%) in the nervous system after KT, followed by nervous system CMV infection (38%) and stroke (5%). Nevertheless, due to the inconsistencies in the types of NCs included and the follow-up time, our results might only serve as an epidemiological reference for the specific incidence differences.

## 1. Introduction

Kidney transplantation (KT) is the preferred option for end-stage renal disease (ESRD), and it contributes to improving patient survival and quality of life compared with hemodialysis [1]. In terms of long-term benefits, KT is the most cost-effective method in renal replacement therapy. However, due to lack of self-care knowledge and poor treatment compliance, patients face challenges after discharge, resulting in increased risks of readmission for KT recipients and undermining patients' safety [2]. Neurological complications (NCs), classified as central nervous system complications and peripheral nervous system complications, are common complications after KT, mainly including cerebrovascular events (stroke and reversible encephalopathy syndrome), central nervous system infections, and metabolic encephalopathy. The long-term cumulative incidence of NCs is up to 85% [3]. Moreover, it is divided into short-term complications (<3 months) and long-term complications (≥3 months). The incidence of stroke after kidney transplantation is about 8%, which is associated with a history of hypertension, diabetes, and atherosclerosis. The incidence of central nervous system infection after renal transplantation is 5–10%, and the fatality rate is up to 75%. Systemic symptoms are usually absent in central nervous system infections and may lead to death in the event of aggravation. The 5-year survival after KT is as high as 90%, but the incidence of NCs after kidney transplantation remains a real concern. NCs after kidney transplantation are attributed to multiple factors, such as infection, hypoxia, metabolism, electrolyte disturbance, posttransplant rejection, and application of immunosuppressants [4]. In recent years, with the development of traditional Chinese medicine (TCM) theory and practice, TCM also plays an important role in improving the gastrointestinal function of patients after KT, with regulating qi and collaterals as the main therapeutic principles.

The article "The Prevalence of Neurological Complication after Renal Transplantation" was retracted in 2023. Reasons: unreliable results or conclusions; concerns about the data; concerns about the peer review; concerns about the citations.

NCs following KT are associated with reduction or withdrawal of immunosuppressive agents and further lead to renal transplant rejection, resulting in a physical and psychological impact on patients and tremendously compromising the prognosis of KT recipients [5]. Nervous system infections are common NCs after KT, and cytomegalovirus (CMV) infection is dominantly responsible for infection after KT. CMV infection, with a strong association with the use of immunosuppressive agents, is a major predisposing factor for acute rejection and is a key influencing element of the survival of recipients [6]. In order to further clarify the incidence and types of NCs after KT, this study conducted a meta-analysis of the published literature on NCs after KT, with the aim of enhancing the understanding of NCs after KT and improving the benefits for KT patients.

## 2. Search Strategy and Selection Criteria

### 2.1. Literature Retrieval

A broad literature search in PubMed, Embase, and Cochrane-Library was performed from inception to December 31, 2021. The searching terms were “renal transplantation” or “kidney transplantation” or “renal transplant” or “kidney transplant” and “complications.” The language was set to English, and references of the included literature were searched and retrospectively added to potentially missing studies whenever possible.

The article "The Prevalence of Neurological Complication after Renal Transplantation" was retracted in 2023. Reasons: unreliable results or conclusions; concerns about the data; concerns about the peer review; concerns about the citations.

### 2.2. Inclusion and Exclusion Criteria of Literature

#### 2.2.1. Literature Inclusion Criteria

The inclusion criteria are as follows. Type of study: retrospective study or randomized controlled clinical trial; study population: postoperative NCs after KT; inclusion of the proportion of patients with NCs and the incidence of NCs; and scientific and standardized research design and clear inclusion criteria and complete data.

#### 2.2.2. Literature Exclusion Criteria

The exclusion criteria are as follows: case reports, failure to obtain a total number of patients and number of patients with target outcome, nervous system adverse reactions or with neurological dysfunction before KT surgery, the number of included participants is less than 10, and repeated study.

#### 2.2.3. Screening of Included Literature

The data were searched by two researchers and Endnote was used for literature management. The duplicate literature was eliminated, and preliminary screening was conducted, respectively. The screening was performed from three levels of article title, abstract, and full text, and then, decisions were made according to the above criteria. The Newcastle–Ottawa scale was used to evaluate the quality of the included literature. In the case of disagreement, the decision on whether to include or not was determined by a third investigator independently. Regarding different articles published with the same study content, only the latest published articles were included.

### 2.3. Data Extraction

The data were extracted and organized by two researchers independently, including authors, publication time, study population type, and research type. Among them, the total number of patients and the number of target outcomes were used as the main effect sizes of the meta-analysis.

### 2.4. Risk of Bias

The studies included in the present meta-analysis were observational studies, randomized controlled studies, and retrospective studies. The purpose of the analysis was to evaluate the epidemiological characteristics of NCs after KT. The following items were used for evaluation with “yes,” “no,” and “unclear” as answers using the evaluation criteria recommended by the Agency for Healthcare Research and Quality (AHRQ) [7]. Is the source of data (survey/literature review) clear? Is the inclusion and exclusion criteria of the exposed and nonexposed groups (or cases and controls) listed or referenced to previous publications? Is the time period for identifying the patient given? If not from human population, is the study subject continuous? Do the evaluators' subjective factors mask other aspects of the research subjects? Are any assessments performed for quality assurance (such as testing/retesting of the primary outcome) described? Are the reasons for excluding any patients from the analysis explained? Are the measures on how to evaluate and/or control confounding factors described? If possible, are strategies on how missing data are handled in the analysis explained? Whether the response rate of patients and the completeness of data collection are summarized. If there is a follow-up, whether the expected percentage of incomplete patient data or follow-up results is identified.

The article "The Prevalence of Neurological Complication after Renal Transplantation" was retracted in 2023. Reasons: unreliable results or conclusions; concerns about the data; concerns about the peer review; concerns about the citations.

### 2.5. Statistical Analysis

The R software meta-package was used to organize and analyze the data. First, the heterogeneity of the included studies was evaluated by the *I*^2^ test. If *I*^2^ = 0, *P* > 0.1 in the two subgroups, it means that there is no heterogeneity in the included studies, and the fixed effect model is used for analysis. If *I*^2^ > 0, *P* > 0.1 in the two subgroups, it means there is heterogeneity, and a random-effects model is used for analysis.

## 3. Results

### 3.1. Results of the Literature Search and Intervention Studies

Our search had 326 citations, which were initially screened on the abstract level for eligibility. After excluding duplicate literature, abstracts, and reviews, 267 pieces of literature were excluded and 59 were included. After being retrieved and reviewed in full text, 17 articles including 11119 patients were considered eligible. This included 3 studies that recorded unclassified NCs (249 participants), 6 that recorded nervous system CMV infection (1489 participants), 3 that recorded headache (243 participants), and 5 that recorded cerebrovascular events (9138 participants). The quality of the included literature met the criteria of AHRQ. Results of the literature search are given in Table 1, and the quality evaluation is shown in Figure 1.

### 3.2. Forest Plot of NCs Incidence

Of the included studies, 3 articles documented unclassified NCs during follow-up, including headache, anxiety and depression, tremor, encephalopathy, and diabetic peripheral neuropathy. In the analysis of the incidence of unclassified NCs in all subjects, there was significant heterogeneity within the group (*I*^2^ = 91%, *p* < 0.01). The random-effects model was used, and the incidence was 0.29, 95% CI (0.16–0.48), as shown in Figure 2.

Of the included studies, 6 articles documented the incidence of CMV infection in the nervous system during follow-up. In the analysis of the incidence of CMV infection in all subjects, there was significant heterogeneity within the group (*I*^2^ = 97%, *p* < 0.01). The random-effects model was used, and the incidence was 0.38, 95% CI (0.26–0.52), as shown in Figure 3.

The article "The Prevalence of Neurological Complication after Renal Transplantation" was retracted in 2023. Reasons: unreliable results or conclusions; concerns about the data; concerns about the peer review; concerns about the citations.

Of the included studies, 3 articles documented the incidence of headache during follow-up. In the analysis of the incidence of headache in all subjects, there was significant heterogeneity in the group (*I*^2^ = 75%, *p*=0.02), and the random-effects model was used, and the incidence rate was 0.55, 95% CI (0.44–0.66), as shown in Figure 4.

Of the included studies, 5 articles documented the incidence of stroke during follow-up. In the analysis of the incidence of stroke among all subjects, there was significant heterogeneity within the group (*I*^2^ = 97%, *p* < 0.01). The random-effects model was used, and the incidence was 0.05, 95% CI (0.02–0.09), as shown in Figure 5.

### 3.3. Publication Bias Analysis and Sensitivity Analysis

Egger's test was used to analyze the publication bias of the included literature, and the results are shown in Figure 6. Statistics were *t* = 0.34, *p*=0.7890 for the meta-analysis of incidence of unclassified NCs; *t* = 0.73, *p*=0.5079 for the meta-analysis of incidence of CMV infection, *t* = 1.01, *p*=0.4954 for the meta-analysis of incidence of headache, and *t* = 0.77, *p*=0.4965 for the meta-analysis of stroke incidence. There was no significant publication bias in the included literature in each group analysis. The sensitivity of the included studies was analyzed by the method of exclusion one by one, and the studies in each group had good stability, as shown in Figure 7.

## 4. Discussion

In this study, the NCs analysis was divided into 4 groups, namely, unclassified NCs (all NCs patients included in the follow-up period), CMV infection, headache, and stroke. Incidence of unclassified NCs was 0.29 (95% CI (0.16–0.48)), of nervous system CMV infection was 0.38 (95% CI (0.26–0.52)), of headache was 0.55 (95% CI (0.44–0.66)), and of stroke was 0.05 (95% CI (0.02–0.09)). It was found that CMV infection has the highest incidence, followed by unclassified, headache, and stroke. Theoretically, the incidence of unclassified NCs should be greater than the sum of the other three, but it ranked second in this study. An in-depth interpretation of the literature shows that the definitions and diagnostic methods for NCs vary in different studies. In the studies of unclassified NCs, no patients with CMV infection were reported, which may be related to the lack of CMV testing; the proportion of headache was significantly lower than that of headache, which might be associated with the distinctive definitions of headache; only one article reported a stroke incidence rate of 2.27% [8], which was not significantly different from the stroke group, and the other two reported no stroke. Therefore, due to the inconsistency in the definitions and detection methods of complications, only the incidence after intragroup meta-analysis is significant, while intergroup comparison results are considered of no statistical significance.

The article "The Prevalence of Neurological Complication after Renal Transplantation" was retracted in 2023. Reasons: unreliable results or conclusions; concerns about the data; concerns about the peer review; concerns about the citations.

The use of immunosuppressive agents is utilized to prevent acute rejection of KT. Posttransplant immune monitoring and optimization of immune regulation contribute to the prediction of impending transplant rejection and avoidance of renal biopsy [9]. However, the drug toxicity and long-term immunosuppression compromise the survival of KT patients. Research has demonstrated that immunosuppressants have a direct or indirect impact on the nervous system, induce neurotoxicity, or increase the risk of central nervous system infection, and the long-term cumulative incidence of NCs after KT is as high as 85% [10]. It has also been found that cyclosporine (CsA), tacrolimus (Tac, FK506), corticosteroids, and muromonab-CD3/Orthoclone (OKT3) are closely associated with posttransplant NCs [11]. In addition to the potential negative impacts of immunosuppression, renal function impairment is also considered a major cause of NCs. For instance, creatinine, eGFR, serum nitrogen, CRP, 1,25-(OH)2D3, intact parathyroid hormone (iPTH), and changes in phosphorus metabolism are associated with psychological and cognitive impairment after KT [12].

In the present study, the incidence of CMV infection was as high as 38% (95% CI: 26–52%). CMV infection is a key contributor to death in KT recipients and is related to long-term chronic graft failure. Therefore, the implementation of effective and timely prevention and treatment of CMV infection after KT is a key to enhancing transplantation outcomes [13]. CMV is a common pathogen in human virus infection and a weak pathogenic factor with mild virulence in individuals with normal immunity. However, CMV is latent in the host for life once infected. When the immune function declines, patients are susceptible to new CMV infection. Stroke is a cerebrovascular circulation disorder caused by cerebrovascular pathological changes, constituting a part of cerebrovascular disease. A study by the American Nephrology Data Statistical System showed that the cumulative incidence of stroke at 3 years after KT receptor surgery was 6.8% [14], and the stroke incidence in this study was 5% (95% CI: 2–9%). We speculated that it correlates with the irreversible effects of end-stage renal disease on the vascular system. In addition, the long-term use of immunosuppressants has a role in the metabolism of glucose and lipids, and the incidence of stroke is inevitably higher than that of ordinary people despite the restored renal function after transplantation. In the present study, the incidence of headache was 55% (95% CI: 44–66%), and immunosuppressants CsA, FK506, and sirolimus were considered the main causes of headache, and it is related to vascular endothelial dysfunction caused by immunosuppressive agents that trigger brain microvascular cells to produce excessive nitric oxide.

The article "The Prevalence of Neurological Complication after Renal Transplantation" was retracted in 2023. Reasons: unreliable results or conclusions; concerns about the data; concerns about the peer review; concerns about the citations.

## 5. Conclusion

Neurological complications yield a high prevalence after renal transplantation. Headache had the highest incidence in the nervous system after KT (55%), followed by nervous system CMV infection (38%) and stroke (5%). Nevertheless, due to the inconsistencies in the types of NCs included and the follow-up time, our results might only serve as an epidemiological reference for the specific incidence differences.

## Figures and Tables

**Figure 1:** Risk assessment chart of included literature.

**Figure 2:** Forest plots of the uncategorized neurological complications meta-analysis.

**Figure 3:** Forest plots of the CMV + meta-analysis.

**Figure 4:** Forest plots of the headache meta-analysis.

**Figure 5:** Forest plots of the stroke meta-analysis.

**Figure 6:** Egger's funnel plot of the publication bias.

**Figure 7:** Forest plots of sensitivity analysis.

**Table 1:** Basic information of enrolled literatures.

Number	First author	Year	Study type	Total cases	Complication types	Complication cases
1	Jehn U [15]	2020	Retrospective	723	CMV	182
2	Moura LR [8]	2015	Review	209	CMV	145
3	Posadas Salas MA [16]	2013	Post hoc analysis	187	CMV	43
4	Mayer G [17]	1988	Retrospective	120	CMV	40
5	Hemmersbach M [18]	2019	Retrospective	166	CMV	85
6	Jarque M [19]	2020	Prospective	84	CMV	26
7	Kateryna K [20]	2014	Retrospective	73	All	28
8	Yardimci N [21]	2008	Retrospective	132	All	18
9	Cengiz N [22]	2015	Retrospective	44	All	19
10	Maggioni F [23]	2009	Retrospective	83	Headache	37
11	Viticchi G [24]	2019	Retrospective	50	Headache	35
12	Viticchi G [25]	2021	Retrospective	110	Headache	59
13	Huang ST [26]	2019	Retrospective	4635	Stroke	146
14	Findlay MD [27]	2016	Retrospective	956	Stroke	26
15	Oliveras A [28]	2003	Retrospective	403	Stroke	19
16	Weng SF [29]	2019	Retrospective	2908	Stroke	79
17	Marchiori PE [30]	2005	Retrospective	236	Stroke	46

## Data Availability

The datasets used during the present study are available from the corresponding author upon request.
